# Image Segmentation under the Optimization Algorithm of Krill Swarm and Machine Learning

**DOI:** 10.1155/2022/8771650

**Published:** 2022-03-24

**Authors:** Qiang Geng, Huifeng Yan

**Affiliations:** ^1^School of Big Data & Software Engineering, Chongqing College of Mobile Communication, Chongqing 401520, China; ^2^Chongqing Key Laboratory of Public Big Data Security Technology, Chongqing 401420, China; ^3^School of Software Engineering, Chongqing University of Posts and Telecommunications, Chongqing 400065, China

## Abstract

This study aims to improve the efficiency and accuracy of image segmentation, and to compare and study traditional threshold-based image segmentation methods and machine learning model-based image segmentation methods. The krill herb optimization algorithm is combined with the traditional maximum between-class variance function to form a new graph segmentation algorithm. The pet dataset is used to train the algorithm model and build an image semantic segmentation system. The results show that when the traditional Ostu algorithm performs image single-threshold segmentation, the number of iterations is about 256. When double-threshold segmentation is performed, the number of iterations increases exponentially, and the execution time is about 2 s. The number of iterations of the improved Krill Herd algorithm in single-threshold segmentation is 6.95 times, respectively. The execution time for double-threshold segmentation is about 0.24 s. The number of iterations is only improved by a factor of 0.19. The average classification accuracy of the Unet network model and the SegNet network model is 86.3% and 91.9%, respectively. The average classification accuracy of the DC-Unet network model reaches 93.1%. This shows that the proposed fusion algorithm has high optimization efficiency and stronger practicability in multithreshold image segmentation. The DC-Unet network model can improve the image detail segmentation effect. The research provides a new idea for finding an efficient and accurate image segmentation method.

## 1. Introduction

With the popularization and development of artificial intelligence (AI), computer vision (CA), as a branch of machine learning, gradually attracts the attention of scholars and has made many achievements [1]. It is to process the collected images or videos to obtain the correct information. In the study of CV-related technologies, the study on image segmentation technology is also listed as one of the key points. Without correct segmentation, there is also no correct image recognition, target detection, and scene analysis. Therefore, the study on image segmentation has great significance for image processing and analysis [2].

The research on image segmentation methods can be divided into two aspects. One is the traditional image segmentation method, and the other is the image segmentation method based on machine learning (ML). The traditional image segmentation methods are mainly based on the segmentation methods of threshold, region, edge, and specific theory. Most of the traditional image segmentation methods are simple and effective, and are used to obtain the main features of the image and improve the efficiency of image analysis and processing. Therefore, scholars have also studied and improved the traditional image segmentation methods. As ML is used more widely and great achievements are made, researchers try to introduce ML into image processing. As a new research direction of ML, deep learning (DL) is used in the field of image analysis and processing. In recent three years, the AlexNet network designed by Hinton and his student Alex Krizhevsky won the championship with an error rate of 15.3% (26.2% of the second) in the ImageNet image recognition competition, which caused a huge response and opened the exploration and research of the convolutional neural network (CNN) on image processing. Fully convolutional networks (FCNs) are applied to image segmentation based on DL.

At present, most of the research on image segmentation is mainly in the medical field. However, the scenes where the image is made are diversified, and these models will have many limitations in practical applications. Therefore, the image segmentation technology is extended from the medical field to others. The swarm intelligence optimization algorithm is combined with the traditional image threshold segmentation algorithm to improve the efficiency of image segmentation. Based on DC-Unet, a semantic segmentation system is constructed to be applied to most images. The swarm intelligence optimization algorithm is used to segment the threshold-based image, and the application of DC-Unet to image segmentation is studied. The effectiveness of these two methods in image segmentation is verified by experiments, and the efficiency and accuracy of image segmentation are further improved. The study provides a direction for exploring an image segmentation method that can be applied to all images.

## 2. Literature Review

### 2.1. Application Status of Machine Learning Algorithms in Image Segmentation

Wang et al. used a multimodal image fusion model based on the maximum energy region to fuse rich information from different modalities in the image fusion stage [3]. In 2018, they mentioned two automatic remote sensing image interpretation methods based on the multiparadigm collaborative framework, which can guide the image segmentation process after the image is classified [4]. Xu et al. proposed an improved fuzzy C-means algorithm for image segmentation. The algorithm combines the neighborhood correlation model with the reliability measure to describe the spatial relationship of the target, thereby improving the robustness and accuracy of the clustering algorithm. The improved algorithm can make up for the defect that the known correlation algorithm is sensitive to noise [5]. Zhang et al. proposed a biogeography-based optimization (BBO) algorithm to find a better clustering solution and applied fuzzy C-means (FCM) to each iteration to make the segmentation effect better [6]. Azimbagirad and Junior proposed a new generalized entropy and studied its application in image segmentation. They use the critical point of Tsallis entropy to tune the precision of each parameter [7].

### 2.2. Application Status of Deep Learning Neural Networks in Image Segmentation

On this basis, Kar et al. discussed deep learning-based semantic segmentation techniques. This technique uses the deep neural network structure to segment images and discusses the basic theory related to deep learning methods used in semantic segmentation [8]. Chen et al. proposed the DeepLap model, which is applied to the cavity convolution in diffusion-convolutional neural networks (DCNNs), and combined with the conditional random field (CRF) to overcome the shortcomings of DCNNs. One is image resolution compression caused by the maximum pooling and downsampling operation, and the other is that the accuracy of the model is affected by the invariance of spatial transformation, making the obtained probability diagram vague [9].

In the field of image segmentation, the latest hot research points focus on machine learning algorithms and deep learning neural networks in the field of artificial intelligence. This provides a crucial theoretical basis for the selection of this research method.

## 3. Research Methods

Swarm intelligence optimization algorithm (SIOA) is a random search algorithm that uses groups to observe the behavior of a certain group and individual behavior, and define the evolution of the group and the specificity of behavior. Then, by simulating the swarm behavior of natural organisms, its properties are studied to solve the swarm optimization problem. The more famous SIOAs are genetic algorithm (GA), particle swarm optimization (PSO), and so on. The krill herd algorithm (KHA) and common machine learning models such as linear models, kernel methods, and support vector machines, decision trees and boosting, and neural network models are all closely related to SIOA. They interact with each other and can do more with less.

### 3.1. Image Segmentation Based on Krill Herd Optimization Algorithm

#### 3.1.1. KHA

Each krill in the krill population will be affected by food and the surroundings during the movement to the food. In KHA, each krill is supposed to be a solution in the connection space and food to be the optimal solution. Under the comprehensive influence of food and surroundings, the information of the krill is updated iteratively and finally the food is found; that is, the global optimal solution is output.

In KHA, the position movement of each krill *i* contains three parts, and the *k*-th movement, *X*_*i*_(*k*), can be expressed as

(1) $$\begin{array}{c} X_{i}\left(k\right)=N_{i}\left(k\right)+F_{i}\left(k\right)+D_{i}\left(k\right). \end{array}$$

In equation (1), *N*_*i*_(*k*) represents the movement of *i* guided by the other krill, known as guided movement. *F*_*i*_(*k*) represents the movement under the influence of food, which is called foraging movement. *D*_*i*_(*k*) represents the random diffusion.

First, guiding the movement. For krill *i*, the *k*-th movement, *N*_*i*_(*k*), can be defined as

(2) $$\begin{array}{c} N_{i}\left(k\right)=N_{\max}a_{i}\left(k\right)+w_{n}N_{i}\left(k-1\right), \end{array}$$

where *N*_max_ is the maximum guided velocity, *N*_*i*_(*k* − 1) is the previous guided movement, *w*_*n*_ ∈ [0,1] is the inertia weight of the two guided movements before and after, and *a*_*i*_(*k*) is the guided movement source, which are defined as

(3) $$\begin{array}{c} a_{i}\left(k\right)=a_{i}^{\text{local}}\left(k\right)+a_{i}^{\text{target}}\left(k\right), \end{array}$$

where *a*_*i*_^local^(*k*) represents the local influence of the neighboring krill on krill *i*, and *a*_*i*_^target^(*k*) represents the guidance of the target direction generated by the optimal krill in the current population.

Second, foraging the movement. It is divided into food guidance and foraging experience. For krill *i*, its *k*-th foraging movement, *F*_*i*_(*k*), is expressed as

(4) $$\begin{array}{c} F_{i}\left(k\right)=v_{f}\beta_{i}\left(k\right)+w_{f}F_{i}\left(k-1\right), \end{array}$$

where *v*_*f*_ is the foraging speed, *F*_*i*_(*k* − 1) is the last foraging movement, *w*_*f*_ ∈ [0,1] is the inertia weight of two foraging movements before and after, and *β*_*i*_(*k*) is the source of foraging movement, which can be defined as

(5) $$\begin{array}{c} \beta_{i}\left(k\right)=\beta_{i}^{\text{food}}\left(k\right)+\beta_{i}^{\text{best}}\left(k\right), \end{array}$$

where *β*_*i*_^food^(*k*) represents the food attraction perceived by krill *i*, and *β*_*i*_^best^(*k*) represents the attraction of the optimal fitness degree obtained by *i* from the initial iteration to the current.

Third, in the KHA algorithm, the diffusion of krill individuals is random, expressed by the following equation:

(6) $$\begin{array}{c} D_{i}\left(k\right)=D_{\max}\delta_{i}\left(k\right), \end{array}$$

where *D*_max_ represents the maximum diffusion velocity, *δ*_*i*_(*k*) represents the current random direction vector, and each term is a random number between [−1,1].

In the KHA algorithm, the effect of guiding movement and foraging movement gradually decreases with the increase of iteration times, and the krill swarm is also constantly approaching the optimal solution. The better the position of the krill is, the smaller the random diffusion should be. Therefore, the number of iterations is added to show a linear decline in the random diffusion of krill individuals, that is,

(7) $$\begin{array}{c} D_{i}\left(k\right)=D_{\max}\left(\frac{1-k}{K}\right)\delta_{i}\left(k\right), \end{array}$$

where *K* is the maximum iteration times.

#### 3.1.2. Improvement of the Krill Herd Optimization Algorithm

The improved krill herd algorithm (IKHA) is studied further, hoping to improve the convergence speed and accuracy of IKHA. Adhvaryyu, et al. proposed IKHA to avoid the algorithm falling into local optimum in iteration and improve its convergence speed and accuracy [10].

In KHA, inertia factors *w*_*n*_ and *w*_*f*_ of induced motion and foraging motion will be larger to avoid the algorithm falling into the minimum, which can improve the global search ability of the algorithm. *w*_*n*_ and *w*_*f*_ can be adjusted to a smaller value to improve the local observation ability of the algorithm in the current location. It is found that the most important thing to improve the performance of the algorithm is to reasonably take the values of *w*_*n*_ and *w*_*f*_. The method for improving the convergence speed and convergence accuracy of KHA is

(8) $$\begin{array}{c} w_{n}=w_{f}=\frac{xs\;d\left(i,j\right)+w_{\min}-w_{\max}}{K}\left(K-k\right), \end{array}$$

where *xs*  *d*(*i*, *j*) ∈ (0,1) represents the similarity of individuals *i* and *j*, *k* represents the current number of iterations, *K* represents the maximum iteration times, *w*_max_ represents the maximum value of induced inertia factor and foraging inertia factor, and *w*_min_ represents their minimum values. This method can adjust the values of the*w*_*n*_ and *w*_*f*_ algorithm according to different krill populations and improve the global search and local exploration abilities of the algorithm. However, in practical applications, this algorithm has weak local exploration ability at the initial iteration and poor global search ability at the end of iteration. This is easy to make the algorithm miss the global optimal solution at the initial iteration and have the optimal value at the end of iteration. In this case, a nonlinear decreasing strategy based on time changing is suggested as follows:

(9) $$\begin{array}{c} w_{n}=w_{f}=w_{\min}\cdot \text{rand}+\left(w_{\max}-w_{\min}\right)\left(2-e^{\log\left(2\right)\cdot k/\text{MI}}\right), \end{array}$$

where *k* represents the current iteration times, and MI represents the current maximum iteration times. When rand ∈ [0,1], *w*_max_ represents the maximum of the induced inertia factor and the foraging inertia factor, and *w*_min_ represents their minimum values. This equation can reduce the values of *w*_max_ and *w*_min_ so that the current search ability can be effectively adjusted in the whole optimization process, the local optimal value is avoided, and the attractive factors of the current global optimal individual to the individual optimization process are increased. The optimization of IKHA is as follows:

(10) $$\begin{array}{c} X_{i}\left(k+\Delta k\right)=X_{i}\left(k\right)+\Delta k\frac{\text{d}X_{i}}{\text{d}k}+r_{1}\left(X_{\text{best}}\left(k\right)-X_{i}\left(k\right)\right), \end{array}$$

where *X*_best_(*k*) is the current global optimal individual, and *r*_1_ is the attraction factor.

#### 3.1.3. Design of Image Segmentation Based on IKHA

IKHA is used to find the best threshold and combined with the maximum between-cluster variance algorithm to study its application in image segmentation.

The flowchart of image segmentation based on IKHA is shown in Figure 1.

In Figure 1, firstly, the grayscale pixel probability is calculated. Meanwhile, the algorithm parameters are set. Initial krill population and individual fitness values are calculated. The current position of the krill individual after the change is calculated. Next, the fitness of the krill population is updated. Once the maximum number of iterations is reached, and the grayscale image is segmented. The segmented image is obtained.

The effectiveness of IKHA in finding the optimal value is realized by segmenting the image and comparing with other algorithms.

### 3.2. Image Segmentation Based on DL

The method of image segmentation based on IKHA and the maximum between-cluster variance algorithm is suitable for gray images with large difference between the target and the background. It is simple, fast, and practical when segmenting these images. However, this segmentation method is not ideal for complex images. The introduction of DL improves the effectiveness of the segmentation of high-dimensional complex images [11, 12]. The image segmentation system based on the DC-Unet network model of DL is studied, and it is introduced from the structure design, the preparation for training datasets, model construction, and model training.

#### 3.2.1. Structure Design of Image Segmentation System

According to the function, the system is divided into three modules: the preprocessing module, model training module, and image segmentation module. Its structure is shown in Figure 2.

The preprocessing module includes the data input interface, data preprocessing, and simple logical judgment. After the image is preprocessed, the model is trained and the image is segmented. And the system is designed according to the three modules, and the flowchart is shown in Figure 3.

It is assumed that the data received by the preprocessing module can be divided into image data and video data. The video data need to be converted into image data. Then, the training model should be judged. If it is the training model, the data should be enhanced. If not, the image data are segmented in the image segmentation module.

#### 3.2.2. Preparation of the Training Dataset

In DL, a large number of data should be input into the dataset to obtain data features and make the model more representative. However, in actual engineering tasks, the datasets for model training are not sufficient sometimes. In this case, the data should be preprocessed to expand the training dataset. After some transformation, the process of generating new data from the original dataset is data enhancement [13]. For image datasets, data enhancement can be realized by geometric transformations, such as rotation transformation, flip transformation, scaling transformation, and random shear. Among them, two or more are usually combined in practical use [14–16].

#### 3.2.3. Model Building

The architecture of DC-Unet is shown in Figure 4.

The structure of DC-Unet is sequential. The input of each network layer is the output of the upper layer. And the convolution layer, the pooling layer, the transposed convolution layer, and the void convolution layer are constructed, respectively.

#### 3.2.4. Model Training

The parameters should be adjusted constantly to make the output of the model close to the ground truth, which is the training process of the model. In the process, the test sets and training sets should be provided to avoid overfitting [17, 18]. The model training is shown in Figure 5.

In Figure 5, eight images in Oxford-IIIT Pet are restricted for use. The DC-Unet network model is pretrained and then formally trained. The Oxford-IIIT Pet dataset is a pet dataset with 37 categories. There are about 200 images per category. The images vary widely in scale, pose, and lighting. All images have associated breed, head ROI, and ground-truth annotations for pixel-level trigram segmentation.

### 3.3. Evaluation Criteria

#### 3.3.1. Evaluation Methods of Threshold Segmentation Algorithms

The image segmentation algorithm is evaluated by iteration times and execution time. The fewer the iteration times are, the shorter the execution time is, and the higher the efficiency of the algorithm is.

#### 3.3.2. Evaluation Methods of Image Semantic Segmentation Algorithms

In the image semantic segmentation, the segmentation method is evaluated by classification accuracy and the average classification accuracy.

The classification accuracy rate is used to represent the effect of each classification type. The calculation equation is [19–21] as follows:

(11) $$\begin{array}{c} {\text{CA}}_{i}=\frac{|P_{i}\cap {\text{GT}}_{i}|}{\left|{\text{GT}}_{i}\right|}, \end{array}$$

where *P*_*i*_ is a collection of pixels of the *i*-th type in the test set, and GT_*i*_ is a collection of pixels marked as the *i*-th type.

The average classification accuracy is the overall description of all kinds of classification accuracy in the dataset. The calculation equation is

(12) $$\begin{array}{c} \text{CAA}=\frac{1}{n}\sum_{i=1}^{n}{\text{CA}}_{i}, \end{array}$$

where *n* is the number of segmentation types in the dataset, *i* is the *i*-th classification, and CA_*i*_ is the classification accuracy of the *i*-th classification [22, 23].

## 4. Results

1. The Ostu algorithm, the KHA-Ostu algorithm, dynamic adjustment of inertia weight krill herd algorithm (DKHA)-Ostu, and IKHA-Ostu are used to segment eight images. The iteration times and execution time of single threshold and double threshold images are recorded, respectively. The experimental results of iteration times of single threshold images are shown in Figure 6.
2. In Figure 6, the iteration times of KHA-Ostu, DKHA-Ostu, and IKHA-Ostu are much lower than those of Ostu for the single-threshold image segmentation. The iteration times of Ostu for eight images are 256, while those of the other three algorithms are less than 25. The iteration times of IKHA-Ostu are the lowest. The average iteration times of the other three algorithms except Ostu are calculated. The average iteration times of KHA-Ostu is 10.3125, those of DKHA-Ostu is 11.725, and those of IKHA-Ostu is 6.95. It is concluded that IKHA-Ostu is superior to other algorithms in the complexity.
3. The experimental results of the iteration times of double threshold image segmentation are shown in Figure 7.
4. The figure shows that the values by Ostu are much larger than those of the other three algorithms. The iteration times of IKHA-Ostu are lower than those of the other three algorithms. When Ostu is used to segment the image with two thresholds, the iteration times are 256 *∗* 256, which shows an exponential growth compared with the single threshold image segmentation. The average iteration times of KHA-Ostu, DKHA-Ostu, and IKHA-Ostu are 34.3875, 34.9875, and 13.9625, respectively. The effects of the three algorithms are significantly improved for single threshold image segmentation. The effect of KHA-Ostu is improved by about 2.33 times, DKHA-Ostu is improved by 1.98 times, and IKHA-Ostu is improved by about 0.19 times. It is proved that IKHA-Ostu is superior to other algorithms in the complexity when it is applied to dual-threshold image segmentation. With the increase of the number of segmentation thresholds, its advantage to improve the efficiency is more obvious.
5. The execution time of single threshold image segmentation is shown in Figure 8.
6. Figure 8 shows that the execution time of Ostu is lower than that of KHA-Ostu, DKHA-Ostu, and IKHA-Ostu in single threshold image segmentation. The average execution time of the four algorithms is 0.004975 s, 0.0219 s, 0.0251 s, and 0.0153 s, respectively. Because the other three algorithms are introduced into the krill herb algorithm, the krill herb algorithm needs more time in single threshold image segmentation. The execution time of IKHA-Ostu is the lowest among KHA-Ostu, DKHA-Ostu, and IKHA-Ostu.
7. The execution time of double threshold image segmentation is shown in Figure 9.
8. Figure 9 shows that the execution time of Ostu is much longer than that of the other three when in the double threshold image segmentation, and its average value is about 2.00 s. The execution time of IKHA-Ostu is shortest, with an average value of about 0.24 s. The average execution time of KHA-Ostu is about 0.58 s and that of DKHA-Ostu is about 0.61 s. It is proved that the efficiency of IKHA-Ostu is higher than the other three algorithms in the double threshold segmentation.
9. Through the above experimental results, the iteration times and execution time of IKHA-Ostu are better than those of KHA-Ostu and DKHA-Ostu in single and double threshold image segmentation. The execution time of IKHA-Ostu in single-threshold image segmentation is longer than that of Ostu because of the time occupied by IKHA-Ostu. However, the execution time of IKHA-Ostu is significantly better than that of Ostu in double-threshold segmentation. IKHA-Ostu is more practical because images usually have multiple thresholds.
10. DC-Unet is trained using the pet dataset, and the results are compared with those of Unet and SegNet. The results are shown in Figure 10.

Figure 10 shows that DC-Unet has more advantages than the other two network models in classifying the individual or the dataset. For dog images in the dataset, the classification accuracy of Unet, SegNet, and DC-Unet are 85.5%, 91.2%, and 92.3%, respectively. For cat images, the classification accuracy of the three network models is 88.1%, 93.7%, and 94.8%. The average classification accuracy of these three models on the pet dataset is 86.3%, 91.9%, and 93.1%.

The DC-Unet network model has higher values than the other two network models whether it is the correct rate of classification of dog and cat categories, or the average correct rate of classification in the pet dataset. This shows that it can improve the image segmentation effect in image semantic segmentation. This is consistent with the findings of Lopez-Bernal et al.. This study discusses the application of different algorithms to solve three different binary classification problems using three different datasets. Comparisons are made in specific case studies and their performance; it is proved that the optimized performance is the best [24].

## 5. Conclusion

Image segmentation is a branch of image processing. With the development of science and technology, image segmentation is also developing in terms of accuracy, efficiency, and generalization. Here, KHA is improved, and the interclass variance in the maximum interclass variance algorithm is used as the fitness function. The proposed IKHA is applied to image segmentation, and the results are compared with other algorithms, which prove that the proposed IKHA is superior in image segmentation. Then, DC-Unet is built, and the image segmentation system is constructed based on it. The model is trained using the pet dataset, and the segmentation effect of the model is compared with that of SegNet and Unet through experiments. When the traditional Ostu algorithm performs image double-threshold segmentation, the execution time is about 2 s. The execution time of the IKHA for dual-threshold segmentation is about 0.24 s. Compared with the Unet network model and the SegNet network model, the average classification accuracy of the DC-Unet network model is the best, reaching 93.1%. The results show that the system can improve the effect of image segmentation. However, there are also some shortcomings: the proposed IKHA still has a slow convergence speed when applied to image segmentation; when the DC-Unet model performs image segmentation, the segmentation effect of the model is reduced in a complex environment. The image segmentation based on KHA and DC-Unet is studied. KHA can segment simple images, and DC-Unet can segment complex images. The combination of these two methods can achieve efficient and accurate segmentation for most images. The research is to use an algorithm to achieve accurate image segmentation of all images, which is also the focus of follow-up research.

## Figures and Tables

**Figure 1:** Flowchart of image segmentation algorithm based on IKHA.

**Figure 2:** Structure of the image segmentation system.

**Figure 3:** Design of image segmentation system based on DL.

**Figure 4:** Architecture of DC-Unet.

**Figure 5:** Model training of DC-Unet.

**Figure 6:** Experimental results of the iteration times of single threshold segmentation.

**Figure 7:** Experimental results of the iteration times of double threshold image segmentation.

**Figure 8:** Execution time of single threshold image segmentation.

**Figure 9:** Execution time of double threshold image segmentation.

**Figure 10:** Training results of network models using the pet dataset.

## Data Availability

The data used to support the findings of this study are included within the article.
